# An Individualized and Everyday Life Approach to Cognitive Rehabilitation in Schizophrenia: A Case Illustration

**DOI:** 10.1155/2012/928294

**Published:** 2012-09-10

**Authors:** M.-N. Levaux, B. Fonteneau, F. Larøi, I. Offerlin-Meyer, J.-M. Danion, M. Van der Linden

**Affiliations:** ^1^Cognitive Psychopathology Unit, Department of Psychology: Cognition and Behavior, University of Liège, 4000 Liège, Belgium; ^2^Psychiatry Service I, Inserm 666 Unit, 67091 Strasbourg, France; ^3^Cognitive Psychopathology and Neuropsychology Unit, University of Geneva, 1211 Geneva, Switzerland

## Abstract

*Objective*. The effectiveness of an individualized and everyday approach to cognitive rehabilitation for schizophrenia was examined in a case study. *Method*. After cognitive and functional assessment, concrete objectives were targeted for the person's everyday complaints. Strategies were constructed based on an analysis of the cognitive profile, daily life functioning, and processes involved in activities. They included a memory strategy for reading, a diary to compensate memory difficulties, and working memory exercises to improve immediate processing of information when reading and following conversations. Efficacy was assessed with outcome measures. *Results*. The program had beneficial effects on the person's cognitive and everyday functioning, which persisted at a 3-year follow-up. *Conclusion*. Findings provide suggestive evidence that an individualized and everyday approach may be a useful alternative in order to obtain a meaningfully lasting transfer of training to daily life, compared to the nomothetic ones which dominate the field.

## 1. Introduction

Cognitive rehabilitation therapy refers to “a behavioral training based intervention that aims to improve cognitive processes … with the goal of durability and generalization” [1]. Recently, two meta-analyses in schizophrenia [1, 2] revealed that cognitive rehabilitation has a positive, small-moderate effect on overall cognition (resp., 0.41 and 0.45; 0.43 at follow-up [1]), psychosocial functioning (resp., 0.35 and 0.42; 0.37 at follow-up [1]), and symptoms (resp. 0.28 and 0.18; no longer significant at follow-up [1]). Moreover, stronger effects on psychosocial functioning were found when cognitive rehabilitation was provided together with psychiatric rehabilitation [1, 2]. The effect size on functioning was larger in Wykes et al. (.59, [1]) than in McGurk et al. (.47, [2]), while the number of studies both evaluating psychosocial functioning and combining it with cognitive rehabilitation were increased in the recent meta-analysis [1]. The analyses indicated that the studies which did not have a significant impact on functioning were providing cognitive rehabilitation in “stand alone” cognitive programs with no functional interventions [1, 2]. Thus, the combination of cognitive rehabilitation and psychosocial rehabilitation served to significantly enhance the response to cognitive intervention.

Generalization and the ability to produce a meaningfully lasting effect represent two major goals of cognitive rehabilitation. Unfortunately, however, a large number of cognitive rehabilitation studies have overlooked both issues. In terms of the ability to produce a meaningfully lasting effect, Wykes et al. [1] report that only 28% and 30% of studies included in their meta-analysis comprised a follow-up assessment for global cognition and functional outcome, respectively, and only 23% of studies included such an assessment for cognition in McGurk et al. [2]. Moreover, when follow-up periods are included, they are many times limited to only few weeks or months. 

The issue of generalization has also been neglected by studies, yet the ultimate goal of remediating cognitive deficits is not simply to improve cognitive test scores but to generalize improvements to durable real-world application [3]. In Wykes et al. [1], only 48% of studies evaluated psychosocial functioning, and, in McGurk et al. [2], this was only 42%. 

In our opinion, there are at least two major reasons why cognitive rehabilitation, until now, has had a limited effect on functional outcome. First, specific difficulties in patients' everyday lives have not been given the importance they deserve when designing and proposing cognitive rehabilitation programs, yet it is these difficulties that should be the main focus of interventions. Few current cognitive remediation programs take functioning into account in their design. Persons with specific functional difficulties (rather than cognitive difficulties) are included in two of these programs. Among those, the “Thinking Skills for Work program” by McGurk et al. [4, 5] has worked as the primary outcome and combines cognitive and vocational rehabilitation, which consists of comprehensive assessment of obstacles to employment, identification of cognitive and behavioral strengths and weaknesses, provision of restorative and compensatory cognitive remediation strategies that are individualized, tracking of functioning,and full integration of work services so that employment specialist can help the client adapt compensatory strategies learned in the intervention to the specific work place. The “Attention Training” intervention by Silverstein et al. [6] is another example, which is fully integrated into social skills training with the goal of improving social functioning. Second, previous studies and interventional strategies have not taken into account the vast heterogeneity inherent in schizophrenia. Taking both these issues into account will hopefully render cognitive rehabilitation programs even more effective, especially in terms of improvements in psychosocial functioning. 

Thus, in addition to identifying the impaired and preserved cognitive domains in a patient with schizophrenia, it is equally important to define the consequences of the cognitive deficits on daily life activities and to develop ecological rehabilitation strategies (i.e., which can be transferred to real-world situations) based on concrete objectives in daily life. Consequently, the efficacy of a cognitive rehabilitation should be based not only on the results of cognitive measures but also on everyday life measures. Moreover, cognitive rehabilitation programs have generally not focused on the real-world difficulties of persons with schizophrenia, but rather, on patients' cognitive difficulties. This has been based on the supposition that the trained cognitive tasks share some common cognitive processes with daily life activities, such that improvement of performance on a cognitive task will lead to beneficial effects on everyday functioning. However, due to the complex nature of the relations between cognitive and real-life functioning, such an approach might not necessarily lead to a significant improvement in daily life functioning. Therefore, we favor an approach which identifies patients' difficulties on everyday activities and endeavors to understand the nature (cognitive or otherwise) of these difficulties and thus to be able to identify which (cognitive or otherwise) processes to remediate (see [7, 8]). 

Secondly, schizophrenia is unmistakably a vastly heterogeneous disorder (e.g., [9, 10]), but this fact has not been taken into account in most cognitive rehabilitation studies, where the same program is administered to all patients. Detailed analyses of the profiles of persons are not carried out, even though people with schizophrenia clearly differ in terms of the degree and type of their cognitive deficits (e.g., [11, 12]), and on a large number of other dimensions including, for example, difficulties in everyday activities, goals, coping capacities, and environmental contexts. The adoption of a single-case methodology is one manner of taking this heterogeneity into account. Indeed, in light of evidence of the heterogeneity of people with neurological lesions, the neuropsychological literature also advocates the use of a single-case methodology in cognitive rehabilitation [13]. In schizophrenia, this approach was primarily used by Velligan and collaborators [14, 15] who developed a Cognitive Adaptation Training (CAT) that utilizes compensatory strategies and supports (such as pill containers with alarms, organization of belongings, and activity checklists) in the home environment and tailored to the specific cognitive impairments of each participant.

In sum, the beneficial effects of cognitive rehabilitation in schizophrenia could be improved by adopting an approach that individualizes treatment and that directly focuses on decreasing the person's everyday difficulties. For this purpose, we concretely propose four steps. (1) The patient's goals and needs are identified, in addition to specific activities that pose problems in everyday life. This information can be assembled using various methods such as open discussions (e.g., with the patient, the patient's caregivers, the clinical team), observations (e.g., of the patient in various contexts or when performing performance-based tasks of everyday activities), or questionnaires of psychosocial functioning. (2) Detailed evaluations are carried out, which include cognitive assessments of both defective and intact processes and the identification of the optimizing factors (i.e., strategies that may improve or facilitate cognitive performance). (3) Based on these cognitive and functional evaluations, reasons are established as to why the patient might have difficulties in the various everyday activities. (4) Ecological rehabilitation strategies, which are combined and chosen according to the rehabilitation objectives, are then proposed to the patient and a “rehabilitation contract” is mutually agreed upon between the patient, and the mental health professional. Such a contract may include information such as what will be remediated and why, how it will be remediated, and the duration and frequency of sessions. In this approach, the patient's needs are directly addressed in a treatment context, thus undoubtedly increasing intrinsic motivation, which is a central issue in treatment programs [3]. What follows is a description of a case study, which will serve as an illustration of this individualized and everyday life approach to cognitive rehabilitation. 

## 2. Case Illustration

D.S. is a 42-year-old woman without a profession and who lives with her husband. She completed one year of superior studies in chemistry when her first psychotic episode appeared at 22 years of age leading to a diagnosis of paranoid schizophrenia according to DSM-IV criteria. She has had approximately 20 hospitalizations; the last one being approximately two years before the rehabilitation program. During acute phases of the disease, D.S. presented delusions, visual and auditory hallucinations, stereotypies, and obsessions. D.S. was clinically stable for at least six months before the rehabilitation apart from occasionally experiencing auditory hallucinations. At the time of the study, her treatment consisted of two atypical antipsychotics (olanzapine: 2 × 10 mg; quetiapine: 1 × 200 mg) and one benzodiazepine (lorazepam: 1 × 2.5 mg), and she was seen by her psychiatrist about twice a month. 

### 2.1. Daily Functioning Complaints

D.S. expressed a desire to be more autonomous and to not have to rely on her husband all the time. She described a number of difficulties in everyday activities: following and retaining television or radio programs, following and retaining conversations, reading and maintaining text information (e.g., from a book or newspaper), remembering appointments, dates, activities (forcing her to write everything down on sheets of paper in order not to forget). These difficulties had a deleterious impact on her everyday functioning, such as social withdrawal. For instance, D.S. did not dare communicate with others as she feared that she would not be able to follow and understand the discussions. Also, if she constantly asked people to repeat what was said, she feared this will get on peoples' nerves or lead them to suspect that she is insane. 

### 2.2. Pre-Rehabilitation Cognitive Assessment

An extensive cognitive battery was administered to D.S., which covered various aspects of cognitive functioning (see Table 1). A score indicating a deficit was set at <−1.65 for the *z*-score and at <10 for the percentile score (in order to be less strict in comparison to a threshold <1.96 and <5; some scores were presented as *z*-scores and others as percentiles, depending on the given norms for each test). Performance was impaired on working memory tests assessing processing load and updating, while storage was preserved. Analysis of executive functioning revealed deficits related to flexibility and planning, but not inhibition. Performance was impaired on the verbal episodic memory tests, but not on the visual episodic memory test. Performances in divided and sustained attentional functions were all impaired. Processing speed was slow, but not impaired. 

## 3. Treatment Study

### 3.1. Design

The rehabilitation consisted of two 90-minute sessions per week (20 in total) and lasted three months. The intervention plan was designed to evaluate the effect of cognitive rehabilitation on functional targets. For this purpose, outcome measures at two different times were used: pre-rehabilitation and post-rehabilitation assessment. 

### 3.2. Targets and Strategies

Based on an analysis of D.S.'s daily functioning complaints and cognitive assessment, three rehabilitation target objectives were defined to improve her daily life functioning. Rehabilitation strategies were constructed according to processes involved in these target activities, analysis of preserved and impaired processes, and the optimizing factors. 

#### 3.2.1. Macrostructure Use

 Based on cognitive assessment, D.S. presented verbal episodic memory deficits, and in particular encoded text information in an unsystematic way. These impairments could explain difficulties she had in reading and remembering the contents of books or newspapers. In order to improve her memory for texts, a structured encoding strategy was proposed to D.S. This involved extracting the main information of a text in an organized manner, by omitting unimportant details and by highlighting significant elements. This strategy could help D.S. both at encoding and consequently at retrieval of a text (i.e., the use of a macrostructure at retrieval could serve as a cue that elicits recall of the text). 

#### 3.2.2. Working Memory Training

 D.S. also expressed difficulties in following conversations, and TV or radio programs. These difficulties, in addition to difficulties in maintaining information from texts from books or newspapers, could be related to a reduction of working memory resources observed in D.S. Thus, improving D.S.'s capacity to process immediate information in working memory could favor the extraction of main information and the binding between external information and mental representation in reading or conversational activities. Consequently, working memory training was implemented with several processing load and dual-task monitoring exercises. 

#### 3.2.3. Diary Use

 Memory (working and episodic) and planning deficits were observed in D.S., which were implicated in her difficulties to remember and plan everyday activities. Thus, an external aid was proposed to compensate for memory and planning deficits and to decrease the anxiety related to forgetting. A personalized diary was created, which was structured with various headings according to her activities, and was implemented in D.S.'s daily life. 

### 3.3. Tasks and Stimuli 

#### 3.3.1. Macrostructure Use

 The macrostructure consisted of six headings: (1) title; (2) spatial context (where?); (3) temporal context (when?); (4) person(s); (5) facts; (6) results and conclusions. Two types of texts that D.S. had particular difficulties with were chosen by her: chapters from a book and newspaper articles. These texts did not differ according to their difficulty, length, and number of essential information contained in the six headings. In total, 17 chapters and 13 articles were used for the rehabilitation sessions (1 chapter and 1 article per session). They were analyzed in order to extract the total number of essential information contained in each of them and in order to construct a scoring grid (according to the six headings). 

After reading a text, D.S. was asked to complete the various headings of the macrostructure (for an example from a newspaper article, see Table 3). Then, she was asked to read this macrostructure once or twice. Finally, D.S. had to recall the text without using the macrostructure both immediately after the session and in the next session, in order to check for long-term retention of the information. The task lasted about 45 minutes and was realized in 18 rehabilitation sessions.

#### 3.3.2. Working Memory Training

 Several types of working memory exercises (36 in total across 14 sessions) were proposed to D.S. (2 to 4 per session, each exercise lasting about 10 minutes): (1) 10-word reconstruction exercises: a word was orally spelt to D.S. beginning with the last letter and she had to find the correct word; 10-number reconstruction exercises: a series of digits were orally read to D.S. who was then asked to provide the number formed by the digits; the words and numbers were of different lengths (4 to 6 letters; 4 to 5 digits) (1 point for each correct response; maximum score for each task = 15); (2) 3 alphabetical ordination exercises of orally presented words (3 to 4 words) (1 point for each correct response; maximum score = 10); (3) 8 exercises from a Brown-Peterson task: a number of four digits and then three words were read to D.S. who had to repeat the words and then recall the number (1 point for each recalled number; maximum score = 15); (4) 5 exercises from a market task: D.S. received a list containing the price of articles in a market. The name of a person and the purchases (2 to 3 articles) were orally presented to D.S. who had to memorize them and calculate the total price (1 point for each correct response, that is, articles, name of the person, and total price; maximum score = 40 to 50). 

#### 3.3.3. Diary Use

 The diary consisted of four headings based on D.S.'s daily functioning: “important dates” (e.g., doctor appointments), “outings” (e.g., with friends), “shopping list,” and “housework”. On one sheet of the diary representing a week, the four headings were positioned on top horizontally and the days of the week were positioned to the left vertically. 

During the first session, D.S. was taught how to use the diary correctly. Two main objectives were proposed: (1) to gather all the information to be remembered in one place by respecting the headings and (2) to consult this diary at the same time of the day (i.e., morning, midday, and evening). For the following sessions, D.S. was asked to bring her diary with her in order to examine whether it was used in a regular and correct manner in daily life. If this was not the case, a discussion of how to improve diary use followed (e.g., use all the headings, make changes in her diary according to her timetable). In total, interviews concerning diary use were carried out in 10 sessions and lasted about 10 minutes each.

### 3.4. Outcome Measures

Outcome measures (administered before and after the rehabilitation program) consisted of assessing macrostructure use, working memory performance, and diary use (parallel versions of macrostructure use and working memory performance were used in order to minimize practice effects). The Subjective Scale to Investigate Cognition in Schizophrenia (SSTICS, [26]) was also administered before and after the rehabilitation program to obtain an index of the person's subjective cognitive complaints for five cognitive domains (memory, attention, executive function, language, and praxis). Finally, a subjective assessment questionnaire for the three rehabilitation objectives was administered at post-rehabilitation.

## 4. Results

### 4.1. Pre-Rehabilitation versus Post-Rehabilitation Comparison

 The post-rehabilitation results (see Table 1) revealed an improvement (i.e., when a performance previously impaired at pre-rehabilitation is within the norms at post-rehabilitation) in both processing load and the updating component of working memory. There was a decrease in the number of errors for planning abilities. Flexibility remained impaired. Verbal episodic memory showed clear improvement. Divided attention (i.e., number of omissions) improved slightly, but sustained attention remained impaired. Finally, working memory storage improved.

Performance of pre- and post-rehabilitation outcome measures was compared (see Table 2) for macrostructure use, working memory tasks, diary use, and the SSTICS. A statistical analysis using chi-square tests was carried out to compare the scores regarding macrostructure use, working memory tasks, and SSTICS.

#### 4.1.1. Macrostructure Use

 The mean immediate recall percentage for chapters and for articles was calculated. Significant improvements were noted for chapters (*χ* ^2^(1) = 35.17; *P* < .001) and articles (*χ* ^2^(1) = 200; *P* < .001).

#### 4.1.2. Working Memory

 Scores on the word reconstruction task and the number reconstruction task improved significantly (resp., *χ* ^2^(1) = 6.5; *P* = .01; *χ* ^2^(1) = 12.53; *P* < .001). The scores on the Brown-Peterson task did not significantly improve from pre-rehabilitation to post-rehabilitation (*χ* ^2^(1) = .08; *P* = .78). Finally, the market task improved significantly (*χ* ^2^(1) = 56.23; *P* < .001).

#### 4.1.3. Diary Use

 D.S. used the diary and its headings correctly from the first session. After three sessions, D.S. stopped using numerous separate reminders scattered around the house as they were now centralized in her diary, and she consulted it regularly (i.e., morning, midday, and evening).

#### 4.1.4. SSTICS

 The total SSTICS score decreased (nonsignificantly) at post-rehabilitation (*χ* ^2^(1) = 1.79; *P* = .18). The decrease essentially concerned attentional complaints that showed a significant decrease (*χ* ^2^(1) = 28.57; *P* < .001), while memory (*χ* ^2^(1) = .74; *P* = .39) and executive complaints (*χ* ^2^(1) = 1.73; *P* = .19) did not significantly diminish. 

#### 4.1.5. Qualitative Self-Assessment

Based on replies on the subjective questionnaire, D.S. reported that the macrostructure headings helped her “very much” in structuring her thoughts and in concentrating when reading. Moreover, D.S. reported that she spontaneously used the macrostructure procedure. She also mentioned that she found herself talking to people more often and giving responses due to an increased ability to comprehend and follow conversations. When asked whether there was an improvement in attention when watching movies or during conversations, she answered “very much.” The use of the diary helped her to plan her week in a more efficient manner (without forgetting), thus decreasing her anxiety level. She reported being better organized when everything was gathered in one place. Finally, she had the feeling of having made progress and was very satisfied with the rehabilitation.

### 4.2. Follow-Up

A follow-up assessment took place three years after the end of the cognitive rehabilitation. During this period, D.S. remained clinically stable without any hospitalizations. As previously, she continued to see her psychiatrist twice a month, and her treatment consisted of two atypical antipsychotics (olanzapine: 2 × 7.5 mg; quetiapine: 2 × 300 mg) and one benzodiazepine (lorazepam 1 × 2.5 mg). Moreover, she did not take part in any kind of rehabilitation (cognitive rehabilitation, cognitive-behavioral therapy, etc.) during this follow-up period. 

Assessments carried out at the follow-up were the same as those for pre- and post-rehabilitation. The results of the follow-up cognitive assessment (see Table 1) indicated that the post-rehabilitation improvements in both processing load and the updating component of working memory, planning, and divided attention remained stable at follow-up. Flexibility remained impaired. Scores for verbal episodic memory, which revealed a general improvement after rehabilitation, indicated no change at follow-up. Finally, her performance in sustained attention remained impaired.

Performance on pre-rehabilitation and follow-up baseline measures were compared (see Table 2) for macrostructure use, working memory tasks, and the SSTICS.

#### 4.2.1. Macrostructure Use

The same types of texts (book chapter and newspaper article) as those used for pre- and post-rehabilitation were administered: one chapter from another book of the same author and one new article.

**Pre-Rehabilitation versus Follow-Up**

Significant improvements on immediate recall scores for the chapters and the articles persisted (for chapters: *χ* ^2^(1) = 9.68; *P* = .002; for articles: *χ* ^2^(1) = 110.08; *P* < .001).

**Qualitative Analysis**

D.S.'s recalls (immediate and delayed) were structured according to the various macrostructure headings and respected the chronological order of the events.

#### 4.2.2. Working Memory Training

The same tasks as those carried out at pre- and post-rehabilitation were administered albeit parallel versions (i.e., different materiel) were used in order to minimize test-retest effects.

**Pre-Rehabilitation versus Follow-Up**

The significant post-rehabilitation improvement disappeared for the word reconstruction task (*χ* ^2^(1) = 2.92; *P* = .087) and for the number reconstruction task (*χ* ^2^(1) = .53; *P* = .47). On the contrary, scores on the Brown-Peterson task significantly improved (*χ* ^2^(1) = 7.99; *P* = .005), and the significant improvement on the market task persisted (*χ* ^2^(1) = 14.86; *P* < .001).

#### 4.2.3. Diary Use

D.S. reported that the regular use of her diary helped her to better memorize her fixed appointments and that she continued to centralize all the important information in one place. Moreover, she has created another diary where she noted (every evening), on the day page, the activities realized during the day in order to have a better awareness of past personal events. 

#### 4.2.4. SSTICS

**Pre-Rehabilitation versus Follow-Up**

The significant decrease after rehabilitation concerning attentional complaints persisted (*χ* ^2^(1) = 42.42; *P* < .001). Stable scores were noted on the total score (*χ* ^2^(1) = .81; *P* = .37) and specifically for memory complaints (27/44 versus 27/44) and executive complaints (*χ* ^2^(1) = 1.55; *P* = .21).

#### 4.2.5. Qualitative Self-Assessment

The same subjective questionnaire as the one used at post-rehabilitation was administered at follow-up. First, D.S. noted that the use of the macrostructure still helped her “very much” to structure her thoughts when reading. When asked whether there was an improvement in attention when watching movies or during conversations, she answered “moderately,” explaining that she followed the news on the TV better but experienced some difficulties in concentrating during longer activities, which could be due to objective deficits in attentional functions. She indicated that the use of the diary had calmed her down because she no longer had to worry about forgetting important events, therefore allowing her to think about other things. She also expressed that she is more autonomous in her daily-life and that she is still very satisfied with the work realized during the cognitive rehabilitation program. 

## 5. Discussion

Despite numerous appeals in the literature for developing other methodological approaches to cognitive rehabilitation research and practice and in light of findings revealing that “stand alone” cognitive rehabilitation programs have not hitherto succeeded in improving patients' everyday functioning in a significant and durable manner, many studies continue to adopt the same approach. Yet, a change is unmistakably needed. In particular, we call for an individualized and everyday life approach to cognitive rehabilitation in schizophrenia in order to attain this goal. In order to do so, a number of issues need to be addressed and carried out in future studies. In particular, specific and crucial difficulties in patients' everyday lives should be the focus of rehabilitation programs. The vast heterogeneity inherent in schizophrenia must also be considered in forthcoming interventions. It has been argued that taking both these issues into account will result in more effective intervention programs in their ability to provide improvements in patients' psychosocial functioning.

The present case study wished to provide an example of how to work within an individual and everyday life approach to cognitive rehabilitation in schizophrenia. In particular, the study showed that it had a beneficial effect on D.S.'s everyday functioning. The efficacy of the rehabilitation program was especially demonstrated based on results from outcome measures. Furthermore, the beneficial effect of the cognitive rehabilitation program was transferred to the person's daily life, as disclosed in her responses to self-assessment questionnaires and subjective reports. Thus, D.S. became autonomous in the application of strategies learned during the rehabilitation program. Indeed, for instance, she spontaneously used the macrostructure procedure and expressed the fact that this strategy helped her to retain more information when reading texts. D.S. also mentioned that the use of her diary allowed her to plan her week in a more efficient manner without forgetting events and furthermore helped decrease her level of anxiety. D.S. also reported an improvement in attention when watching movies or when following conversations and discussions. This resulted in D.S. talking to people more often, compared to before the cognitive rehabilitation program. Finally, D.S. reported less attentional complaints in her daily life. 

The meaningfully lasting beneficial effects were largely evident in that they were still present when pre-rehabilitation and follow-up scores were compared. However, for some of these measures, significant post-rehabilitation improvement disappeared after the 3-year period. These results suggest that the meaningfully lasting effects were less robust for rehabilitation targets that were not directly associated with compensatory interventions that D.S. still used at the follow-up assessment and/or that rehabilitation sessions aimed at refreshing acquisition would have been necessary. Moreover, D.S. had transferred the learned strategies to her daily-life on a long-term basis: she continued to employ her diary in an efficient manner and continued to structure her reading according to the macrostructure headings. Thus, compensatory approaches, which teach a strategy, have showed to produce life-long changes in function as long as the intervention is effective and the person continues to use the compensatory strategy. Additionally, D.S. expressed being more organized and autonomous—two crucial goals of any rehabilitation program. 

In sum, the originality and interest of this study was to take into account the various complaints that a person diagnosed with schizophrenia experienced in her daily life and to use these as rehabilitation objectives. Different rehabilitation strategies were implemented for each of the complaints, and they were adapted according to her cognitive profile. These elements undoubtedly contributed to the fact that the cognitive rehabilitation program was well accepted by D.S. Thus, an individualized and everyday life approach appears to be an effective alternative to improving the effects of cognitive rehabilitation on both cognitive and daily life functioning in people with schizophrenia. Furthermore, these benefits were shown to be maintained at long-term follow-up.

Some limitations of the study should be mentioned. Firstly, there are limits related to an ABA design (A: outcome measures; B: intervention), which are less capable of establishing a causal relation. However, a protocol with multiple outcome measures or other designs (e.g., type ABAB) was not possible to implement for practical reasons: such a protocol requires numerous assessments and, consequently, is very tiresome and tedious for the patient and such protocol is difficult to design, especially when ecological measures are involved. Moreover, the quality of the case study would have been improved with the inclusion of measures defining the severity of psychiatric symptoms pre- and post-rehabilitation. This will be taken into account in future cognitive rehabilitation studies.

Finally, it is also important to underline that the other psychological dimensions (such as auditory hallucinations, obsessional symptoms, social anxiety), which had an impact on D.S.'s everyday functioning, would also have been important to take into account in the individualized rehabilitation program in order to further increase its efficacy. Indeed, cognitive functioning is by far not the sole factor involved in functional outcome in schizophrenia. Fett et al. [27], in their meta-analysis examining relations between cognitive functioning (both neurocognitive and social cognitive) and functional outcome in patients with nonaffective psychosis, found that cognitive functioning explains 25% of the variance of functional status of patients with schizophrenia, and thus as much as 75% of the variance in outcome was left unexplained. There are at least two implications related to this finding. First, it is necessary that other factors significantly related to functional outcome be identified. Secondly, intervention programs must integrate strategies that remediate and improve these additional areas. Indeed, as observed in Wykes et al. [1] and McGurk et al. [2], cognitive rehabilitation approaches clearly need to be combined with other forms of intervention in order to maximize their impact on functional outcome. Studies have shown that a number of other factors are also significantly related to functional outcome in patients with schizophrenia. These factors include (but are not limited to) symptomatology (especially negative symptoms; [28]), various psychological processes such as social cognition [29], dysfunctional attitudes [30], metacognitive processes [31], poor insight [32], and finally environmental factors, such as family attitudes [33], negative stereotypes [34], and internalized stigma [35]. 

Therefore, we advocate an individualized, integrative, and everyday rehabilitation approach, which includes interventional strategies that help improve, in addition to cognitive factors, other factors that also play a significant role in functional outcome in schizophrenia. Further, we propose to carry out multidimensional evaluations, which include not only cognitive and functional assessments, but also comprise a large array of other dimensions. This integrative approach is important to take into account as schizophrenia is a disorder that affects many different areas and levels of functioning. Moreover, these areas are complementary and interdependent. That is, patients will have difficulties in a number of different areas (e.g., cognitive, motivational,affective) at the same time, and one area may have an impact on the other (e.g., motivational problems may negatively affect affective and cognitive functioning). 

## Figures and Tables

**Table 1:** Pre-rehabilitation, post-rehabilitation, and follow-up cognitive assessment.

Cognitive tests	Pre-rehabilitation	Post-rehabilitation	Follow-up
*Working memory*			
Storage			
(i) Digit span (forward) (MEM-III)	−0.7	0.49	−0.7
Processing load			
(i) Digit span (backward) (MEM-III)	−1	0.76	0.17
(ii) Number of trials for digit span (MEM-III)	**−2.33**	0.33	−0.33
(iii) Letter-number sequencing (MEM-III)	−1.33	−0.66	−0.66
Updating			
(i) Working memory (TAP): median RT/SD RT/omission(s)	P84/P50/**P4**	P79/P50/P18	P76/P50/P18
*Executive functions*			
Inhibition			
(i) Go/no-go (TAP): median RT/SD RT/error(s)	P14/P27/P<46	**P1**/P38/P42	P34/P46/<P42
Flexibility			
(i) Flexibility (TAP): median RT/SD RT/error(s)	–P10/**P7**/P27	**P7/P2**/P82	P12/P16/**P8**
(ii) Verbal fluency: phonological/semantic	−0.33/−1.42	0.18/**−2.37**	0.16/−0.71
Planning			
(i) Six Elements Test: total score/error(s)	−1.48/−1.5	**−2.62**/−0.08	0.01/0.32
*Episodic Memory*			
Explicit verbal episodic memory*			
(i) Logical memory (MEM-III): (I) First recall/total recall/	−1.33**/−1.67**	/	/
learning curve/theme	−1/−1	/	/
(II) Total recall/retention%/theme	**−1.67**/−1/−1	/	/
(ii) California Verbal Learning Test:			
First recall A/fifth recall A/total recall A/	**−1.93**/**P5-25/−2**	0.2/P50/−0.91	/
Short-term recall A/cued recall A	−1.6**/−1.67**	−0.44/−1.2	/
Delayed recall A/delayed cued recall A	**−2/−2.42**	−1.62/−1.49	/
Recognition/false recognition	**P5-25**/**P5-25**	P50/**P5-25**	/
(iii) RL/RI-16: immediate recall/free recall I/cued recall I	/	/	P99/−1.5/P99
Free recall II/cued recall II	/	/	**−1.84**/P25
Free recall III/cued recall III	/	/	−1.57/P99
Delayed free recall/delayed cued recall/recognition (/16)	/	/	**−3.6/P5-25**/16
Explicit visual episodic memory			
(i) Face recognition (MEM-III): part I/part II/retention	0.33/−0.33/−0.67	/	/
*Attentional functions*			
Divided attention			
(i) Divided attention (TAP): median RT/SD RT/omission(s)	P62/P42/**P4**	P38/P14/P12	P76/P16/<P18
Sustained attention			
(i) Digit continuous ordination: mean efficiency: 0–10 min/	**−2.62**	**−2.76**	**−2.83**
10–20 min/0–20 min	**−2.72/**−**2.82**	**−2.72/−2.79**	**−3.22/−3.1**
*Processing speed*			
(i) Digit symbol—coding (WAIS-III)	−1	−0.67	−0.33

*Different episodic memory tests were used at different moments of evaluation (pre-rehabilitation, post-rehabilitation, follow-up) in order to avoid learning effects; numbers in bold indicate a deficit score (< −1.65 for the *z*-scores, <10 for the percentiles); RT: reaction time; SD: standard deviation; digit span, letter-number sequencing, logical memory (MEM-III; [16]); working memory, go/no-go, flexibility, divided attention (TAP; [17]); digit symbol (WAIS-III; [18]); verbal fluency [19]; Six Elements Test ([20]; French adaptation, [21]); California Verbal Learning Test ([22]; French adaptation, [23]); RL/RI-16 [24]; digit continuous ordination [25].

**Table 2:** Pre-rehabilitation, post-rehabilitation, and follow-up outcome measures.

Outcome measures	Pre-rehabilitation	Post-rehabilitation	Follow-up
*Macrostructure use *			
(i) Chapter: mean immediate recall percentage	40	81^∗a^	62^∗b^
(ii) Article: mean immediate recall percentage	0	100^∗a^	71^∗b^
*Working memory *			
(i) Word reconstruction task: correct response (/16)	6	9^∗a^	8
(ii) Number reconstruction task: correct response (/20)	7	12^∗a^	8
(iii) Brown-Peterson task: correct response (/64)	36	37	48^∗b^
(iv) Market task: correct response (/60)	13	45^∗a^	29^∗b^
*SSTICS *			
(i) Total score (/84)	59	51	54
(ii) Memory complaints score (/44)	27	24	27
(ii) Attentional complaints score (/20)	20	15^∗a^	13^∗b^
(iv) Executive complaints score (/12)	8	7	9

^∗a^Significant effect for pre-rehabilitation versus post-rehabilitation comparison; ^∗b^significant effect for pre-rehabilitation versus follow-up comparison.

**Table 3:** Example of macrostructure training for a newspaper article entitled “Oil, the luxury product.”

Title: oil, the luxury product	
Spatial context (where?): in the world, and in Belgium	
Temporal context (when?): present day	
Person(s): OPEP or the Organization of Petroleum Exporting Countries	
Facts: the increase of oil price creates an important world problem. This is due to the fact that China buys oil so that there is no competition and, moreover, the capacities of refining are decreasing	
Results and conclusions: in Europe, the European Commission is revising its forecasts (less oil production)	
